# Gujiansan Ameliorates Avascular Necrosis of the Femoral Head by Regulating Autophagy via the HIF-1*α*/BNIP3 Pathway

**DOI:** 10.1155/2021/6683007

**Published:** 2021-08-31

**Authors:** Jie Han, Yuan Chai, Xiao-yun Zhang, Feng Chen, Zhi-wei Xu, Zhe Feng, Qian Yan, Shuai-bo Wen, Yu-kun Wu

**Affiliations:** Department of Orthopedics, Ruikang Hospital Affiliated with Guangxi University of Chinese Medicine, Nanning 530011, China

## Abstract

**Background:**

Clinically, the traditional Chinese medicine compound Gujiansan has been widely used in the treatment of steroid-induced avascular necrosis of the femoral head (SANFH). The present study aimed to investigate the mechanisms underlying the therapeutic effect of Gujiansan.

**Methods:**

A rat model of SANFH was established by the injection of dexamethasone (DEX) at a high dosage of 25 mg/kg/d. Then, Gujiansan was intragastrically administered for 2 weeks, 4 weeks, and 8 weeks, and histological examination of the femoral head was performed. The expression levels of related mRNAs and proteins were analyzed by qRT-PCR, Western blotting, and immunohistochemistry, and the levels of bone biochemical markers and cytokines were detected with ELISA kits.

**Results:**

Gujiansan administration ameliorated SANFH and induced the expression of hypoxia-inducible factor-1*α* (HIF-1*α*), Bcl-2/adenovirus E1B 19 kDa interacting protein 3 (BNIP3), LC3, and Beclin-1 in the rat model in a dose- and time-dependent manner, and Gujiansan promoted osteocalcin secretion at the femoral head. In addition, Gujiansan increased the levels of bone formation- and bone resorption-specific markers (osteocalcin (OC), bone-specific alkaline phosphatase (BAP), tartrate resistant acid phosphatase-5b (TRACP-5b), N-terminal telopeptides of type I collagen (NTX-1), and C-terminal telopeptide of type I collagen (CTX-1)) and decreased the levels of proinflammatory cytokines (TNF-*α*, IL-6, and CRP) in a dose- and time-dependent manner.

**Conclusions:**

Gujiansan accelerates the formation of a new bone, promotes the absorption of the damaged bone, inhibits the inflammatory response, induces autophagy of the femoral head via the HIF-1*α*/BNIP3 pathway, and ultimately ameliorates SANFH.

## 1. Introduction

Avascular necrosis of the femoral head (ANFH) is one of the most common osteoarthritic diseases worldwide. Currently, over 30 million people suffer from ANFH globally, including more than 8 million individuals in China [1, 2]. In particular, since the development of hormone drugs and their wide application, the incidence of steroid-induced avascular necrosis of the femoral head (SANFH) has gradually increased, and it frequently occurs in patients receiving high-dose steroid treatment, including patients with systemic lupus erythematosus [3]. Clinically, Western medicine mainly adopts conservative treatment, which cannot delay or reverse the progression of SANFH. When the femoral head collapses, surgical treatment is often used. The service life of joint prostheses is limited, and it is difficult to avoid postoperative revision and secondary prosthesis replacement [4]. Delaying or reversing the progression of SANFH have always been challenges in clinical treatment.

Traditional Chinese medicine has received increasing recognition and been a subject of in-depth pharmacological research for the treatment of osteoarthritic diseases [5, 6]. Icariin (derived from plants of the genus *Epimedium*) can accelerate fracture healing via activation of the WNT1/*β*-catenin osteogenic signaling pathway [7]. Antler extract exerts a positive curative effect on ANFH by promoting osteoblastic proliferation through the regulation of cell cycle progression [8]. Intravenous infusion of cervus and cucumis polypeptides relieves pain and improves hip function in subjects with ANFH [9]. Jiangu decoction (which includes *Astragalus*, *Drynaria fortunei*, and *Salvia miltiorrhiza*) is effective in inhibiting femoral head adipogenic differentiation and decreasing peroxisome proliferator-activated receptor (PPAR) levels to prevent and treat SANFH [10]. Compound Danshen (which includes *Astragalus*, icariin, and *Salvia miltiorrhiza*) exerts favorable preventive effects on bone loss through the promotion of osteogenesis and inhibition of osteoclast bone resorption [11]. Chengzai Wan (including *Astragalus* and antler) promotes the function of L-type voltage-sensitive calcium channels in osteoblasts pretreated with methylprednisolone [12]. The Chinese medicine compound Gujiansan, which was developed by the Ruikang Hospital Affiliated with Guangxi University of Chinese Medicine, contains the main active ingredients of the compound medicines described above and has been clinically used to treat thousands of patients with SANFH, but its pharmacological mechanism is still unclear.

Studies have shown that autophagy may be related to the development of bone diseases, and the regulation of the p62 levels by autophagy is important for bone formation [13]. Hypoxia-induced autophagy requires the hypoxia-inducible factor-1*α* (HIF-1*α*) dependent Bcl-2 adenovirus E1a 19 kDa interacting protein 3 (BNIP3), and it is involved in the removal of mitochondria during the autophagic response [14]. Knockdown of HIF-1*α* or BNIP3 expression obviously abrogates the activation of hypoxia-induced autophagy and the enhancement of osteoclastogenesis, and suppression of autophagy significantly attenuates osteoclast differentiation under hypoxic conditions [15]. Although the pathogenesis of SANFH is not well known, ischemia/hypoxia is the fundamental cause of SANFH, and ischemia/hypoxia-induced autophagy participates in the progression or repair of SANFH [16, 17].

Therefore, we hypothesized that Gujiansan might regulate mitochondrial autophagy via the HIF-1*α*/BNIP3 signaling pathway and ultimately improve femoral head necrosis. In this study, we first established a rat model of femoral head necrosis and then administered Gujiansan to ultimately reveal the mechanisms underlying the therapeutic effect of Gujiansan in SANFH.

## 2. Experimental

### 2.1. Animals and Drugs

A total of 120 adult Wistar rats (male : female ratio, 1 : 1; weight, 280–330 g; age, 6 months) were purchased from the Medical Laboratory Animal Center of Guangdong Province. The rats were housed in a temperature-controlled environment (25°C ± 2°C) with a 12-hour light/dark cycle and were given free access to food and water. The experimental studies were approved by the Institutional Animal Care and Use Committee of Ruikang Hospital Affiliated with Guangxi University of Chinese Medicine (Approval No: DW-20200118-003). Gujiansan is a solid phase powder that contains 100 g of American ginseng (*Panax quinquefolius* L.), 50 g of taizi ginseng (*Pseudostellaria sylvatica* (Maxim.) Pax), 100 g of *Astragalus* (*Astragalus membranaceus* Fisch. ex Bunge), 30 g of deer antler (Cornu cervi Pantotrichum), 50 g of Tian Qi (*Panax notoginseng* (Burkill) F.H.Chen), 50 g of *Drynaria fortunei* (*Davallia mariesii* H.J.Veitch), 30 g of *Ganoderma* (*Ganoderma lucidum* Karst), 50 g of *Salvia miltiorrhiza* (*Salvia miltiorrhiza* Bunge), 50 g of Qianjinpa (*Flemingia philippinensis* Merr. et Rolfe), 50 g of douchi ginger (*Lonicera japonica* Thunb.), 30 g of inner gold (Galli gigeriae endothelium corneum), 30 g of *Asarum* (*Asarum sieboldii* Miq.), 10 g of saffron (*Crocus sativus* L.), and 50 g of smilax (*Acorus calamus* L.). The abovementioned Chinese herbal medicines were purchased from and identified by the Department of Pharmacy, Ruikang Hospital Affiliated with Guangxi University of Chinese Medicine. These medicines were ground into powders and combined according to the amounts described above by Xiaoyun Zhang, Feng Chen, and Zhi-wei Xu for use in the animal experiments.

### 2.2. Modeling of Femoral Head Necrosis and Treatment

A rat model of SANFH was established by injection of dexamethasone (DEX, Sigma, China) [18]. SANFH development was induced in rats by intramuscular injection of 25 mg/kg DEX weekly for 8 weeks. Equivalent volumes of phosphate-buffered saline (PBS) were injected as the control at the corresponding time points (control group). After 8 weeks of intramuscular injection, the rats were subjected to digital radiography (DR) examination (Goodsee, #GDA32-02, China) of the femoral head.

After establishing the SANFH model, the rats were randomly divided into five groups: the model group (gavaged with 1 ml saline), pravastatin group (gavaged with 4 mg/kg pravastatin in 1 ml saline, Bristol-Myers Squibb, #C14200165411, China) [17], low-dose group (L-Gujiansan, gavaged with 1 g/kg Gujiansan in 1 ml saline), medium-dose group (M-Gujiansan, gavaged with 2 g/kg Gujiansan in 1 ml saline), and high-dose group (H-Gujiansan, gavaged with 4 g/kg Gujiansan in 1 ml saline). Six rats were included in each group. The intragastric treatments described above were administered once a day for 2 weeks, 4 weeks, and 8 weeks. All the rats were given free access to food and water. The doses of Gujiansan (1 g/kg, 2 g/kg and 4 g/kg) were chosen based on clinical experience, preliminary experiments in rats, and common methods of dose translation between species [19]. Pravastatin has been demonstrated to be useful in preventing steroid-induced ONFH in animal models [17, 20], so we selected pravastatin as the positive control.

### 2.3. Sampling Methods

After treatment with Gujiansan for 2 weeks, 4 weeks, and 8 weeks, the rats were first subjected to DR examination of their femoral head. Then, the rats were anesthetized using 1% sodium pentobarbital (35 mg/kg per SD rat). Celiac venous blood was immediately harvested and centrifuged at 5000 rpm for 10 min, and the serum was used for ELISA. Then, the rats were sacrificed with excessive anesthesia. The femoral head was harvested for histological examination, qRT-PCR, Western blotting, and immunohistochemistry.

### 2.4. Hematoxylin and Eosin Staining

The femoral head was fixed in 4% paraformaldehyde-PBS solution for 3 days. After decalcification by incubation in EDTA decalcification buffer (BOSTER, #AR1071, China) for 5 days at room temperature, the femoral head was embedded in paraffin and then cut into 5 *μ*m sections. The sections were stained as follows: 70% ethyl alcohol for 10 s, diethylpyrocarbonate-treated water for 5 s, hematoxylin with RNase inhibitor for 20 s, 70% ethyl alcohol for 30 s, and eosin Y in 100% ethyl alcohol for 20 s, followed by dehydration in a series of alcohol concentrations for 30 s each and in xylene for 2 min. Images of H&E staining were captured at 400× magnification (CX71, Olympus Corporation, Tokyo, Japan). Five visual fields were randomly selected from each section to count the chondrocyte number, and the mean was quantified in each subgroup sample.

### 2.5. RNA Preparation and qRT-PCR

The femoral heads were placed in liquid nitrogen and ground, and then, the total RNA was extracted using TRIzol reagent (Invitrogen, CA, USA). cDNA was synthesized using a cDNA Synthesis Kit (Takara, Dalian, China). Quantitative RT-PCR (qRT-PCR) was performed to measure mRNA expression levels using SYBR Green and a LightCycler 480 detection system (Roche Diagnostics, Indianapolis, USA). GAPDH mRNA expression levels were used for normalization. The primer sequences are given in Table 1. The qRT-PCR results were analyzed and expressed as relative mRNA levels based on the CT value, and the relative expression levels were converted to fold change.

### 2.6. Western Blotting Assay

The femoral heads were placed in liquid nitrogen and ground and then lysed using lysis buffer. The total protein concentrations of the lysates were measured using a micro-BCA protein assay kit (Pierce, Rockford, IL, USA). The samples were separated with 12% SDS-polyacrylamide gels and then electrophoretically transferred to polyvinylidene difluoride membranes. After blocking in 5% nonfat milk solution for 1 h, the membranes were incubated with anti-HIF-1*α* (Abcam, ab179483, USA, dilution 1 : 500), anti-BNIP3 (Abcam, ab109362, USA, dilution 1 : 500), anti-Beclin-1 (Abcam, ab207612, USA, dilution 1 : 500), anti-LC3 (CST, 3868s, USA, dilution 1 : 500), and anti-GAPDH antibodies for 2 h at 37°C. Then, the membranes were washed three times and incubated with horseradish peroxidase-conjugated secondary antibodies at room temperature for 1 h. Next, the membranes were treated with ECL solution (Millipore, Darmstadt, Germany) and imaged. The gray values of each protein band were measured with Photoshop CS5 software (Adobe, San Jose, CA, USA). The relative band intensities were assessed as the ratio of the gray value of each protein band to that of the corresponding GAPDH band.

### 2.7. Immunohistochemistry Assay

After decalcification, the femoral heads were embedded in paraffin and then cut into 5 *μ*m sections. After hydration and blocking, the slides were treated with peroxide. An antiosteocalcin antibody (Abcam, ab13420, USA, dilution 1 : 500) was added to the slides and incubated at 37°C for 2 h. After incubation with a secondary antibody at 37°C for 1 h, the slides were treated with 3,3′-diaminobenzidine (DAB) solution. Finally, the slides were lightly counterstained with hematoxylin and dehydrated. Visual analysis was performed with an Olympus fluorescence microscope (Olympus, CX71, Japan) at 400× magnification. The medium optical density (MOD) of osteocalcin expression in each group was analyzed by Image-Pro Plus software (Media Cybernetics, USA).

### 2.8. ELISA

A rat OC ELISA kit (Cloud-Clone Corp, #SEA471Ra, China), rat BAP ELISA kit (Jiancheng, #A059-1, China), rat TRACP-5b ELISA kit (Cloud-Clone Corp, #SEA902Ra, China), rat NTX-1 ELISA kit (Cloud-Clone Corp. #CEA639Ra, China), rat CTX-1 ELISA kit (Cloud-Clone Corp, #CEA665Ra, China), rat interleukin-2 (IL-2) ELISA kit (CUSABIO, #CSB-E04628r, China), rat tumor necrosis factor-*α* (TNF-*α*) ELISA kit (CUSABIO, #CSB-E11987r, China), rat interleukin-6 (IL-6) ELISA kit (CUSABIO, #CSB-E04640r, China), and rat C-reactive protein (CRP) ELISA kit (CUSABIO, #CSB-E07922r, China) were used to measure the concentrations of bone formation- and bone resorption-specific markers and cytokines in this study. All the assays were performed strictly following the manufacturer's instructions.

### 2.9. Statistical Methods

The data were statistically analyzed using SPSS 17.0 (SPSS Inc., Chicago, IL). All the results are presented as the mean values ± standard deviations. ^*∗*^*P* < 0.05,  ^*∗∗*^*p* < 0.01 , and ^*∗∗*^*p* < 0.001 were considered statistically significant. Statistically significant differences between groups were determined by Student's *t*-test. Multiple comparisons were made among ≥3 groups using 1-way ANOVA followed by the Bonferroni post hoc test. The nonparametric Mann–Whitney *U* test was used if data were not normally distributed. Figures were graphed using GraphPad Prism 5 (GraphPad Software, USA).

## 3. Results

### 3.1. Gujiansan Ameliorates SANFH

DR examination of the femoral head showed early osteonecrosis in the rat SANFH model, and the necrotic area was predominantly located in cancellous bone and the chondral region. In the SANFH model, the femoral head exhibited shrinkage and partial collapse, and the bone trabeculae appeared thinner. After 2, 4, and 8 weeks of L-, M-, and H-Gujiansan administration, necrosis of the femoral head was partially repaired in a dose- and time-dependent manner. After 8 weeks of H-Gujiansan administration, the cartilage layer and bone trabecula appeared markedly thicker. DR images (Figure 1) showed that Gujiansan can accelerate the repair of the femoral head.

H&E staining of the chondral region (Figure 2) indicated that the amount of cartilage and the number of chondrocytes were increased in the model group compared to the normal group. After 2, 4, and 8 weeks of L-, M-, and H-Gujiansan administration, the bone lacuna reduced, the cartilage layer tended to be intact, the cartilage cell capsule had proliferated, and the amount of cartilage and the number of chondrocytes increased in a dose- and time-dependent manner. Importantly, the ratio of eosinophilic chondrocytes to total chondrocytes was increased after Gujiansan or pravastatin administration. H&E staining showed that Gujiansan can induce new bone formation of the femoral head.

DR (Figure 1) and H&E staining (Figure 2) indicated that Gujiansan can induce bone formation and accelerate the repair of the femoral head in a dose- and time-dependent manner.

### 3.2. Gujiansan Activated Autophagy and the HIF-1*α*/BNIP3 Pathway in the Rat SANFH Model

qRT-PCR and Western blotting analyses were used to detect the mRNA and protein expression levels of HIF-1*α*, BNIP3, LC3, and Beclin-1 in the rat SANFH model (Figure 3). Compared with those in the L-Gujiansan group, the levels of HIF-1*α*, BNIP3, LC3, and Beclin-1 in the M-Gujiansan and/or H-Gujiansan groups were significantly increased in a dose-dependent manner. After 2, 4, and 8 weeks of Gujiansan administration, the levels of HIF-1*α*, BNIP3, LC3, and Beclin-1 were increased in a time-dependent manner (*p* < 0.05). These data showed that Gujiansan can activate autophagy and the HIF-1*α*/BNIP3 pathway in a dose- and time-dependent manner.

### 3.3. Gujiansan Regulates the Levels of Bone Formation- and Bone Resorption-Specific Markers and Inhibits the Inflammatory Response

Using commercial ELISA kits, we measured the levels of bone formation- and bone resorption-specific markers. The results in Table 2 provide that at 2, 4, and 8 weeks, the levels of OC, BAP, TRACP-5b, NTX-1, and NCTX-1 in the L-Gujiansan, M-Gujiansan, H-Gujiansan, and pravastatin groups were substantially higher than those in the model group. Surprisingly, compared with those in the L-Gujiansan group, the levels of OC, BAP, TRACP-5b, NTX-1, and NCTX-1 in the H-Gujiansan group were significantly increased in a dose-dependent manner. Compared with those in the corresponding 2-week groups, the levels of OC, BAP, TRACP-5b, NTX-1, and NCTX-1 in the 4/8-week group were significantly increased in a time-dependent manner. In addition, we measured the expression levels of osteocalcin in femoral head sections using an immunohistochemistry assay after 2, 4, and 8 weeks of Gujiansan administration and found that Gujiansan treatment induced osteocalcin expression in a dose- and time-dependent manner (Figure 4).

Furthermore, Table 3 provides that the concentrations of TNF-*α*, IL-6, and CRP were significantly increased, and the concentration of IL-2 was significantly decreased in the model group compared with the normal group. After Gujiansan treatment, the concentrations of TNF-*α*, IL-6 ,and CRP were significantly decreased, and the concentration of IL-2 was significantly increased in a dose- and time-dependent manner.

These data showed that Gujiansan accelerates the formation of new bone, promotes the absorption of damaged bone, and inhibits the inflammatory response in the rat SANFH model, thereby promoting the repair of femoral head necrosis.

## 4. Discussion

The incidence of SANFH has gradually increased because of the wide application of hormone drugs. Steroids are known to inhibit osteogenic differentiation and decrease bone formation in BMSCs while concomitantly inducing steroid-induced avascular necrosis of the femoral head (SANFH) [1]. Therefore, in this study, a rat model of SANFH was established by intramuscular injection of DEX. The homemade traditional Chinese medicine compound Gujiansan contains a variety of active ingredients that are used for the treatment of bone diseases, and Gujiansan has been successfully used in the clinic to treat thousands of patients with SANFH [7–12]. Our team studied the effects of Gujiansan on SANFH in a rat model. Based on common methods of dose translation between species, clinical dose experience, and preliminary experiments in rats, we chose three doses (1 g/kg, 2 g/kg, and 4 g/kg) to perform this study [19]. After the intragastric administration of Gujiansan for 2, 4, and 8 weeks, we found that Gujiansan could increase the expression of bone formation- and bone resorption-specific markers, inhibit the inflammatory response in the serum, and induce the expression of HIF-1*α*, BNIP3, LC3, and Beclin-1 in a dose- and time-dependent manner. In summary, our study showed that Gujiansan has therapeutic effects on SANFH.

Under normal circumstances, bone formation markers (e.g., OC and BAP), bone resorption markers (e.g., NTX-1, CTX-1, and TRACP-5b), and cytokines (IL-2, TNF-*α*, IL-6, and CRP) are expressed at relatively low levels, and they significantly affect the process/repair of SANFH [21, 22]. OC is a secreted osteoblast-specific noncollagenous protein of the bone extracellular matrix that circulates in the blood, and it can partly reflect osteoblastic activity during bone formation [23]. SANFH is often accompanied by chronic inflammation, and traditional Chinese medicine (Shenggu Zaizao pills) can effectively inhibit the levels of proinflammatory cytokines (IL-4, IL-6, and TNF-*α*), which may be one of the therapeutic mechanisms by which traditional Chinese medicine treats SANFH [24, 25]. In this study, we found that Gujiansan could increase the levels of OC, BAP, TRACP-5b, NTX-1, CTX-1, and IL-2 in the serum, decrease the levels of TNF-*α*, IL-6, and CRP, and increase the expression of OC in the bone. These results indicate that Gujiansan can accelerate the formation of a new bone, promote the absorption of the damaged bone, and inhibit the inflammatory response in a rat model of SANFH.

The process of autophagy is controlled by autophagy-related genes and accompanied by an increase in autophagy-related protein expression [26]. The conversion of the soluble form of LC3 (LC3-I) to the autophagic vesicle-associated form (LC3-II) is considered to be a major marker of autophagy [27]. Beclin-1 (also known as Atg6 in yeast) is a core protein essential for autophagy initiation and other biological processes [28, 29]. Under hypoxic conditions, hypoxia-inducible factor-1*α* is involved in various signal transduction pathways. As a target gene that is directly regulated by HIF-1, BNIP3 is an important signaling molecule for hypoxia-induced mitochondrial autophagy and plays an important role in the process of recovery from various diseases [30, 31]. A variety of active ingredients in Gujiansan can regulate the expression of autophagy-related proteins to regulate the process of autophagy. Ginsenosides from ginseng (including American ginseng and Tian Qi) can regulate autophagic activity [32]. *G. lucidum* triterpene extract (GLT) induces the formation of autophagic vacuoles and upregulates the protein expression of Beclin-1 and LC-3 [33]. Tao-Hong-Si-Wu decoction significantly promotes the expression of HIF-1*α* and VEGF in the femoral head tissue of rabbits and markedly inhibits the apoptosis of osteocytes, chondrocytes, and bone marrow cells [34]. In rats with SANFH, Gujiansan increased the levels of HIF-1*α*, BNIP3, LC3, and Beclin-1 in a dose- and time-dependent manner, indicating that Gujiansan could activate autophagy and the HIF-1*α*/BNIP3 pathway in SANFH.

At present, autophagy and bone homeostasis are known to be closely related, and autophagy regulates bone formation and bone resorption [35, 36]. Autophagy and apoptosis are markedly promoted in ANFH bone tissues, and increased TNF-*α* expression regulates osteoblast autophagy and apoptosis via the p38 MAPK/NF-*κ*B signaling pathways [37]. Zhao et al. demonstrated that autophagy regulates hypoxia-induced osteoclastogenesis, and the activation of autophagy under hypoxic conditions is caused by the HIF-1*α*-dependent upregulated expression of BNIP3 [15]. In neurofibromatosis type I (NF1) overexpressing BMSCs, NF1 overexpression promotes new bone formation after fracture by enhancing autophagy and inhibiting mTORC1 signaling, indicating that promoting autophagy can promote new bone formation [38]. Unfortunately, at present, we have not measured the mineral density of the femoral head and more autophagy-related proteins (such as p62); meanwhile, we cannot determine which active ingredients in Gujiansan exert a therapeutic effect on SANFH and which active ingredient or ingredients exert a regulatory effect on autophagy in SANFH. These are the limitations of this study and also our next direction in future studies.

In conclusion, we found that Gujiansan accelerates the formation of a new bone, promotes the absorption of the damaged bone, inhibits the inflammatory response, induces autophagy of the femoral head, possibly via the HIF-1*α*/BNIP3 pathway, and ultimately ameliorates SANFH (Figure 5). Based on these studies and its clinical usage, we believe that Gujiansan may serve as a novel therapeutic drug for SANFH. In the future, our team will explore other relevant molecular mechanisms in depth and carry out clinical research.

## Figures and Tables

**Figure 1:** Gujiansan ameliorating SANFH in rats. Digital radiography (DR) was used to observe the femoral head at the 0 week, 2nd week, 4th week, and 8th week (*n* = 6). Red arrow, normal area. Yellow arrow, lesion area. Gujiansan increased the cartilage layer, and the bone trabeculae appeared thicker; thus, Gujiansan promoted the repair of the femoral head in a dose- and time-dependent manner.

**Figure 2:** Gujiansan promoting the proliferation of chondrocyte cysts and chondrocytes in the rat model of SANFH. (a) H&E staining was used to observe the chondral region of the femoral head. Magnification, 400×. Red arrow, cartilage cell capsule and its encased chondrocytes in the normal cartilage layer. Green arrow, proliferating cartilage cell capsule and its encased chondrocytes. (b) The numbers of chondrocytes in each group and each time point. (1) Normal group. (2) Model group. (3) L-Gujiansan group. (4) M-Gujiansan group. (5) H-Gujiansan group. (6) Pravastatin group. The data are presented as the mean ± SD (*n* = 5). ^*∗*^*P* < 0.05 vs. the normal group. ^#^*P* < 0.05 vs. the model group.

**Figure 3:** Gujiansan activating autophagy and the HIF-1*α*/BNIP3 pathway in the rat model of SANFH. qRT-PCR and Western blotting were performed to detect the mRNA and protein expression levels of HIF-1*α*, BNIP3, LC3, and Beclin-1. GAPDH was used as the control. (1) Normal group. (2) Model group. (3) L-Gujiansan group. (4) M-Gujiansan group. (5) H-Gujiansan group. (6) Pravastatin group. The data are presented as the mean ± SD (*n* = 6). ^*∗*^*P* < 0.05 vs. the normal group. ^#^*P* < 0.05 vs. the model group. ^&^*P* < 0.05 vs. the L-Gujiansan group at the corresponding week. ^▼^*P* < 0.05 vs. the corresponding group at 2 weeks.

**Figure 4:** Gujiansan inducing the expression of osteocalcin in the rat model of SANFH. (a) Immunohistochemistry was used to detect the protein expression of osteocalcin. (b) The MOD of osteocalcin expression was calculated using Image-Pro Plus 6.0 software. (1) Normal group. (2) Model group. (3) L-Gujiansan group. (4) M-Gujiansan group. (5) H-Gujiansan group. (6) Pravastatin group. The data are represented as the mean ± SD (*n* = 6). ^*∗*^*P* < 0.05 vs. the normal group. ^#^*P* < 0.05 vs. the model group. ^&^*P* < 0.05 vs. the L-Gujiansan group at the corresponding week. ^▼^*P* < 0.05 vs. the corresponding group at 2 weeks.

**Figure 5:** Schematic diagram of the mechanism by which Gujiansan regulates SANFH repair.

**Table 1:** Primers used for qRT-PCR analysis.

Gene name	Prime name	Primers (5′ to 3′)	Length
GAPDH	Forward	TGACAACTTTGGCATCGTGG	78
	Reverse	GGGCCATCCACAGTCTTCTG	

HIF-1*α*	Forward	AGCAATTCTCCAAGCCCTCC	91
	Reverse	CGGTGGCAGTGACAGTGAT	

Caspase-3	Forward	TCTACCGCACCCGGTTACTA	88
	Reverse	CGTACAGTTTCAGCATGGCG	

Beclin-1	Forward	CCCAGCCAGGATGATGTCTAC	96
	Reverse	AGTCTCCGGCTGAGGTTCTC	

Bcl-2	Forward	ACTCTTCAGGGATGGGGTGA	94
	Reverse	TGACATCTCCCTGTTGACGC	

BNIP3	Forward	ATTGGTCAAGTCGGCCAGAA	81
	Reverse	TCATGCTGAGAGTAGCTGTGC	

LC3	Forward	TGGTGGAAGAGACGAAAGCC	76
	Reverse	ACCAGCATCGTAGAGGGTCT	

Atg5	Forward	CAAGCAGCTCTGGATGGGAC	140
	Reverse	AAAGGCCGTTCAGTTGTGGT	

P62	Forward	GTGGAACCCCAGTAAGAGGC	115
	Reverse	TGAATACCAGCTGTCCGAGC	

**Table 2:** Concentrations of OC, BAP, TRACP-5b, NTX-1, and CTX-1 in each group on the 2nd, 4th, and 8th weeks (*n* = 6).

Groups	Week	OC (pg/ml)	BAP (ng/ml)	TRACP-5b (ng/ml)	NTX-1 (ng/ml)	CTX-1 (pg/ml)
Normal	2	136.05 ± 3.81	12.50 ± 0.40	4.58 ± 0.21	6.64 ± 1.20	415.40 ± 24.42
	4	133.59 ± 5.67	11.64 ± 0.66	4.90 ± 0.36	7.60 ± 1.22	404.77 ± 25.58
	8	131.55 ± 4.77	12.66 ± 0.83	4.99 ± 0.46	7.80 ± 1.15	428.93 ± 23.21

Model	2	8.78 ± 2.13^*∗*^	0.70 ± 0.41^*∗*^	0.22 ± 0.065^*∗*^	2.98 ± 0.17^*∗*^	152.78 ± 7.81^*∗*^
	4	7.31 ± 2.48^*∗*^	0.76 ± 0.28^*∗*^	0.18 ± 0.041^*∗*^	2.81 ± 0.14^*∗*^	157.25 ± 11.04^*∗*^
	8	10.35 ± 3.31^*∗*^	0.86 ± 0.51^*∗*^	0.20 ± 0.066^*∗*^	2.95 ± 0.19^*∗*^	154.90 ± 10.63^*∗*^

L-Gujiansan	2	22.35 ± 5.46^#^	1.63 ± 0.15^#^	0.42 ± 0.10^#^	3.30 ± 0.073^#^	171.32 ± 4.31^#^
	4	23.50 ± 3.46^#^	2.19 ± 0.59^#▼^	0.72 ± 0.11^#▼^	3.46 ± 0.072^#^	182.30 ± 13.60^#^
	8	26.90 ± 6.84^#▼^	2.35 ± 0.31^#▼^	0.84 ± 0.13^#▼^	3.51 ± 0.15^#▼^	192.53 ± 4.28^#▼^

M-Gujiansan	2	40.58 ± 3.97^#&^	3.03 ± 0.30^#^	0.83 ± 0.12^#&^	3.50 ± 0.11^#&^	201.53 ± 12.10^#&^
	4	40.77 ± 7.07^#&^	3.58 ± 0.57^#&^	1.06 ± 0.26^#&▼^	3.83 ± 0.33^#&^	220.85 ± 11.78^#&▼^
	8	48.06 ± 2.36^#&▼^	3.71 ± 0.27^#&▼^	1.10 ± 0.19^#&▼^	3.83 ± 0.12^#&▼^	225.88 ± 12.96^#&▼^

H-Gujiansan	2	54.33 ± 4.99^#&^	4.16 ± 0.26^#&^	1.51 ± 0.23^#&^	4.24 ± 0.24^#&^	230.83 ± 8.37^#&^
	4	54.22 ± 3.47^#&^	5.07 ± 0.27^#&▼^	1.59 ± 0.18^#&^	4.36 ± 0.47^#&^	241.90 ± 7.60^#&▼^
	8	58.55 ± 4.96^#&▼^	5.11 ± 0.34^#&▼^	1.71 ± 0.24^#&▼^	4.40 ± 0.25^#&^	247.99 ± 11.14^#&▼^

Pravastatin	2	64.76 ± 9.53^#^	6.15 ± 0.69^#^	2.18 ± 0.35^#^	4.68 ± 0.063^#^	261.37 ± 7.17^#^
	4	70.42 ± 10.58^#^	6.17 ± 0.81^#^	2.21 ± 0.19^#^	4.80 ± 0.19^#^	267.53 ± 13.37^#^
	8	72.72 ± 4.22^#▼^	7.09 ± 0.49^#▼^	2.70 ± 0.14^#▼^	5.09 ± 0.13^#▼^	282.93 ± 18.49^#▼^

Data are represented as the means ± SD (*n* = 6). ^*∗*^*P* < 0.05 vs. the normal group. ^#^*P* < 0.05 vs. the model group. ^&^*P* < 0.05 vs. L-Gujiansan corresponding weeks' group. ^▼^*P* < 0.05 vs. corresponding 2 weeks' group.

**Table 3:** Concentrations of IL-2, TNF-*α*, IL-6, and CRP in each group on the 2nd, 4th, and 8th weeks (*n* = 6).

Groups	Week	IL-2 (pg/mL)	TNF-*α* (pg/mL)	IL-6 (pg/mL)	CRP (ng/mL)
Normal	2	40.53 ± 0.96	3.01 ± 0.71	0.28 ± 0.02	22.12 ± 1.88
	4	39.75 ± 1.14	3.29 ± 0.67	0.17 ± 0.084	23.84 ± 1.19
	8	39.84 ± 1.16	2.20 ± 0.61	0.33 ± 0.047	21.75 ± 1.65

Model	2	5.63 ± 0.42^*∗*^	47.31 ± 1.81^*∗*^	1.67 ± 0.078^*∗*^	234.98 ± 5.86^*∗*^
	4	4.46 ± 0.45^*∗*^	50.67 ± 1.79^*∗*^	1.69 ± 0.015^*∗*^	236.28 ± 4.46^*∗*^
	8	3.14 ± 0.34^*∗*^	53.13 ± 1.78^*∗*^	1.79 ± 0.019^*∗*^	244.59 ± 4.83^*∗*^

L-Gujiansan	2	21.73 ± 1.05^#^	25.21 ± 0.99^#^	1.15 ± 0.074^#^	149.95 ± 4.79^#^
	4	22.69 ± 0.89^#^	26.93 ± 0.73^#^	1.08 ± 0.045^#^	136.64 ± 7.75^#^
	8	24.54 ± 0.81^#▼^	22.81 ± 1.04^#▼^	0.99 ± 0.054^#▼^	129.31 ± 7.80^#▼^

M-Gujiansan	2	24.38 ± 1.30^#&^	21.36 ± 1.08^#&^	1.00 ± 0.033^#&^	118.68 ± 7.40^#&^
	4	25.74 ± 0.81^#&^	20.62 ± 0.70^#&^	0.88 ± 0.070^#&^	116.72 ± 3.99^#&^
	8	27.95 ± 1.01^#&▼^	16.12 ± 0.86^#&▼^	0.82 ± 0.063^#&▼^	107.31 ± 3.98^#&▼^

H-Gujiansan	2	29.04 ± 1.43^#&^	16.34 ± 1.03^#&^	0.78 ± 0.078^#&^	90.13 ± 4.08^#&^
	4	29.87 ± 0.71^#&^	14.59 ± 1.17^#&^	0.78 ± 0.050^#&^	88.07 ± 9.99^#&^
	8	31.53 ± 0.75^#&▼^	14.22 ± 1.06^#&▼^	0.60 ± 0.021^#&▼^	71.86 ± 7.53^#&▼^

Pravastatin	2	33.26 ± 1.09^#^	12.21 ± 0.67^#^	0.60 ± 0.033^#^	67.36 ± 5.52^#^
	4	33.36 ± 0.78^#^	9.89 ± 1.04^#^	0.53 ± 0.047^#^	58.33 ± 8.38^#^
	8	35.72 ± 1.04^#▼^	6.17 ± 0.57^#▼^	0.43 ± 0.054^#▼^	50.80 ± 5.76^#▼^

Data are represented as the means ± SD (*n* = 6). ^*∗*^*P* < 0.05 vs. the normal group. ^#^*P* < 0.05 vs. the model group. ^&^*P* < 0.05 vs. L-Gujiansan corresponding weeks' group. ^▼^*P* < 0.05 vs. corresponding 2 weeks' group.

## Data Availability

The data used to support the findings of this study are included within this article.
